RETRACTED

# α2,6-Sialylation mediates hepatocellular carcinoma growth *in vitro* and *in vivo* by targeting the Wnt/β-catenin pathway

**DOI:** 10.1038/oncsis.2017.40

**Published:** 2017-05-29

**Authors:** Y Zhao, A Wei, H Zhang, X Chen, L Wang, H Zhang, X Yu, Q Yuan, J Zhang, S Wang

**Affiliations:** 1 Department of Biochemistry and Molecular Biology, Institute of Glycobiology, Dalian Medical University, Liaoning Province, China; 2 School of Life Science and Medicine, Dalian University of Technology, Liaoning Province, China; 3 Department of Pathology, Dalian Medical University, Liaoning Province, China

## Abstract

Abnormal sialylation due to overexpression of sialyltransferases has been associated with tumorigenesis and tumor progression. Although ST6Gal-I influences cancer persistence and progression by affecting various receptors, the underlying mechanisms and mediators remain largely obscure, especially in hepatocellular carcinoma (HCC). We found that ST6Gal-I expression was markedly upregulated in HCC tissues and cells, high levels being associated with aggressive phenotype and poor prognosis. Furthermore, we examined the roles and mechanisms of ST6Gal-I in HCC tumorigenesis and metastasis *in vitro* and *in vivo*. ST6Gal-I overexpression promoted proliferation, migration and invasion of Huh-7 cells, whereas its knockdown restricted these abilities in MHCC97-H cells. Additionally, in a mouse xenograft model, ST6Gal-I-knockdown MHCC97-H cells formed significantly smaller tumors, implying that ST6Gal-I overexpression can induce HCC cell malignant transformation. Importantly, enhanced HCC tumorigenesis and metastasis by ST6Gal-I may be associated with Wnt/β-catenin signaling promotion, including β-catenin nuclear transition and upregulation of downstream molecules. Together, our results suggest a role for ST6Gal-I in promoting the growth and invasion of HCC cells through the modulation of Wnt/β-catenin signaling molecules, and that ST6Gal-I might be a promising marker for prognosis and therapy of HCC.

## Introduction

Hepatocellular carcinoma (HCC) is the fifth most frequently diagnosed malignant tumor and the second leading cause of growing life-threatening cancer worldwide.^1^ The close correlation between its incidence and the number of deaths attributed to this cancer indicate its high fatality rate. Approximately 80–90% of cases occur in Asia and Africa, and in China, the large majority of which are associated with chronic hepatitis B virus infection.^2, 3^ Currently, most of HCC patients cannot be diagnosed in the early stage and they therefore lost the best opportunity for treatment.^4, 5^ Despite tremendous advances in early diagnosis and surgery, HCC incidence continues to increase worldwide. Demonstrations of the efficacy of targeted molecular therapies have triggered the search for additional molecules capable of improving patient survival.

RETRACTED

Glycosylation is a post-translational modification that affects protein folding, stability and activity, and plays important roles in many biological and pathological processes such as immune recognition and tumor progression.^6, 7^ In cancer cells, normal glycosylation is altered^8^ by various causes such as glycosyltransferase dysregulation, changes in the tertiary conformation of the peptide backbone, and alterations of sugar nucleotide donors and cofactors.^9, 10^ Dall’olio F *et al.*^11^ reported that the expression of glycosyltransferase can be regulated by the genetic and epigenetic changes. Abnormal sialylation is a distinctive feature of tumor cells associated with malignant phenotypes including invasiveness and metastatic potential.^12, 13^ For example, gastric and colorectal cancers present high levels of sialyl-Lewis A (SLe^A^) and sialyl-Lewis X (SLe^X^) as terminal epitopes of protein O-glycans, N-glycans and glycolipids.^14^ There are 20 sialyltransferases to be identified, and they were divided into β-galactoside α2,3-sialyltransferases (ST3GalI–VI), β-galactoside α2,6-sialyltransferases (ST6Gal-I and II), GalNAc α2,6-sialyltransferases (ST6GalNAcI–VI) and α2,8-sialyltransferases (ST8SIAI–VI) families.^15^

It has been reported that the high expression of ST6Gal-I increases in the levels of α2,6-sialylation, and correlates with tumorigenesis and tumor progression.^16, 17, 18^ Lu *et al.*^19^ showed that α2,6-sialylated glycans can promote the malignant phenotypes of many tumors by regulating the related signaling pathways. ST6Gal-I is known to regulate the interaction between galectin-1 and α2,6-sialylated N-glycans, and further prevents angiogenesis and tumor progression.^17, 20, 21^ The Rabinovich lab showed that ST6Gal-I overexpression increased in the α2,6-sialylation levels of glycoproteins, and inhibited the binding of galectin-1 and promoted the cellular apoptosis.^22, 23^ In our previous study, we found that upregulation of ST6Gal-I increased the adhesive capability of mouse hepatocarcinoma cell to lymph node.^24^ However, the predictive and prognostic values of ST6Gal-I and its effect on HCC progression remained unclear.

In this study, we aimed to unravel the functions and mechanisms of ST6Gal-I in modulating the growth *in vitro* and *in vivo* of HCC. Moreover, its association with HCC clinical characteristics and the potential underlying mechanisms were explored. Surprisingly, examination of ST6Gal-I levels in HCC and paired normal samples revealed high expression in the former and a close correlation with survival rate. We found that ST6Gal-I upregulation promoted the proliferation, migration and invasion ability of HCC cells. Furthermore, of the pathways tested, ST6Gal-I had the largest influence on Wnt/β-catenin signaling. Therefore, ST6Gal-I might be a promising marker for prognosis and therapy of HCC.

RETRACTED

## Results

### ST6Gal-I expression is significantly upregulated in HCC tissues and cell lines

To explore the role of ST6Gal-I in HCC development, ST6Gal-I was stained by immunohistochemistry (IHC) in representative pairs of cancerous and matched non-tumor liver sections from HCC patients (Figure 1a). Pearson’s chi-squared test identified a significant correlation between ST6Gal-I expression with patient sex, number of lesions and pathologic grade (Table 1). We found that ST6Gal-I-positive patients experienced poorer 5-year overall survival than ST6Gal-I-negative patients (Figure 1b). Moreover, ST6Gal-I positive expression was found to correlate with a short disease-free survival time (Figure 1c). The results are consistent with ST6Gal-I being a potential biomarker of carcinoma progression.^25, 26^ In HCC and normal liver cell lines, ST6Gal-I was expressed in all tested cells as indicated by qPCR and western blot assays. The highest expression was observed in MHCC97-H cells, compared to which Huh-7 cells exhibited low expression (Figures 1d and e). ST6Gal-I expression and localization were confirmed by confocal microscopy, and the results revealed low ST6Gal-I expression in the latter, but high expression in the Golgi apparatus of the former (Figure 1f).

### ST6Gal-I overexpression promotes Huh-7 cell proliferation, invasion and migration *in vitro*

To investigate its function in HCC, ST6Gal-I was overexpressed by transfecting Huh-7 cells with the recombinant vector pcDNA3.1/ST6Gal-I. Expression of ST6Gal-I at mRNA and protein levels was increased in these cells compared to those transfected with an empty pcDNA3.1 plasmid (mock) and parental cells (Huh-7) (Figures 2a and b). Immunofluorescence demonstrated that compared to the control treatment, overexpression of ST6Gal-I increased its presence in the Golgi apparatus of Huh-7 cells (Figure 2d). In addition, ST6Gal-I overexpression resulted in a significant increase in α2,6-sialylation on Huh-7 cell surface (Figures 2c and e). CCK-8 assay showed that at 24, 48, 72 and 96 h after transfection, ST6Gal-I significantly enhanced cell growth rate (Figure 2f). Cancer cell growth was also assessed by colony formation assay. Huh-7 cells overexpressing ST6Gal-I formed significantly more colonies than control cells (Figure 2g). Accordingly, ST6Gal-I overexpression in Huh-7 cells triggered cell cycle arrest in S phase and a reduction in the number of cells in G0/G1 (Figure 2h). Moreover, the wound closure ability of Huh-7/ST6Gal-I cells was remarkably higher than that of control cells after 0, 4, 8 and 12 h (Figure 2i). Using Transwell/Matrigel assays, we found that *in vitro*, the mobility and invasiveness were dramatically increased in ST6Gal-I-overexpressing cells as compared to control groups (Figures 2j and k). Taken together, these findings suggest that ST6Gal-I functions as an oncogene by promoting cancer cell proliferation.

RETRACTED

### ST6Gal-I knockdown attenuates MHCC97-H cell proliferation, invasion and migration *in vitro*

To further verify the role of ST6Gal-I in HCC, we analyzed the effects of ST6Gal-I knockdown on the malignant phenotypes of MHCC97-H cells. ST6Gal-I mRNA and protein expression in MHCC97-H/shST6Gal-I cells was substantially lower than that in those transfected with the control construct and non-transfected MHCC97-H cells as indicated by qPCR, western blotting and immunofluorescence (Figures 3a). Lectin blotting and flow cytometry assay revealed that ST6Gal-I expression was successfully knocked down in MHCC97-H/shST6Gal-I cells (Figures 3c and e). The growth of MHCC97-H/shST6Gal-I cells was suppressed when compared to the control groups (Figure 3f). Accordingly, in an evaluation of the effects of ST6Gal-I knockdown on clonogenic capacity, colony formation was found to be reduced by shST6Gal-I knockdown (Figure 3g). Scratch assays showed that decreased ST6Gal-I expression significantly attenuated MHCC97-H cell migration (Figure 3i). The proportion of ST6Gal-I knockdown cells in S phase was smaller than that in negative control groups, and lower than the percentage arrested at G1/S (Figure 3h). Correspondingly, measurement of cell motility by Transwell/Matrigel assay revealed that suppression of ST6Gal-I restricted migration of MHCC97-H/shST6Gal-I cells (Figures 3j and k). These findings suggest that ST6Gal-I expression is positively correlated with the proliferation, migration and invasion potential of HCC cells.

### Roles and expression of ST6Gal-I in liver tumorigenicity in mice

To examine the effect of ST6Gal-I on tumorigenesis *in vivo*, nude mice were inoculated with ST6Gal-I-knockdown or control cells. Both tumor size and growth rate were dramatically decreased in the MHCC97-H/shST6Gal-I group (Figures 4a and b). In addition, tumor weights were markedly lower in this group (Figure 4c). The average tumor volume at the injection site 4 weeks after inoculation of ST6Gal-I-knockdown cells was obviously smaller than that in the control group (Figure 4d). ST6Gal-I expression in xenograft tumor tissues was also decreased in the MHCC97-H/shST6Gal-I group (Figures 4e and f). Further, over the course of diethylnitrosamine (DENA)-induced liver tumorigenesis, ST6Gal-I expression was gradually increased, while no apparent changes were observed in the control group (Figures 4g and h). Therefore, ST6Gal-I might be involved in the tumorigenesis and development of hepatocarcinoma.

RETRACTED

### ST6Gal-I overexpression augments Wnt signaling pathways in HCC cells

To explore the possible mechanisms underlying the effects of ST6Gal-I on the malignant behaviors of HCC cells, we analyzed the PI3K/Akt, MAPK and Wnt/β-catenin signaling pathways. The results showed that the expression of p-GSK-3β, β-catenin, Cyclin D1, c-Myc, TCF1 and TCF4 was significantly higher in Huh-7/ST6Gal-I cells than in control cells, while the expression of p-β-catenin and GSK-3β proteins was not changed (Figures 5a and b). Additionally, there were no apparent differences in the expression levels of Erk1/2, p-Erk1/2, JNK and p-JNK in ST6Gal-I-overexpressing compared to control cells (Figures 5c and d). Expression of MMP-2, MMP-7 and MMP-9 was generally higher in ST6Gal-I-overexpressing than in control cells (Figures 5e and f). Moreover, confocal immunofluorescence microscopy showed increased expression and accumulation of β-catenin in the cytoplasm, then β-catenin released into the nucleus (Figure 5g). Together, this indicates that ST6Gal-I overexpression could upregulate the Wnt signaling pathway in HCC cells.

### ST6Gal-I knockdown inhibits Wnt signaling pathway in MHCC97-H cells

Next, we observed that whether the inhibited HCC cell proliferation results from the inhibition of Wnt signaling pathway. We found that the expression of p-GSK-3β, β-catenin and related downstream proteins significantly decreased as a result of reduced ST6Gal-I levels (Figures 6a and b), while there were no apparent changes in the proteins of Erk1/2 and JNK signaling pathways (Figures 6c and d). In addition, ST6Gal-I silencing also decreased the expression of CD147/MMPs (Figures 6e and f). Confocal microscopy revealed that β-catenin was diffusely distributed following ST6Gal-I knockdown, with a lower proportion being found in the nucleus (Figure 6g). These data clearly demonstrate that ST6Gal-I knockdown could inhibit the Wnt signaling pathway in HCC cells.

### The effects of ST6Gal-I on the Wnt signaling pathway in mice

From the above results, we have found ST6Gal-I knockdown inhibited Wnt signaling in MHCC97-H cells and the tumorigenicity in xenograft mice. Here, western blot analysis of Wnt signaling in xenograft tumor tissues showed significantly decreased expression of the Wnt signaling molecules in the ST6Gal-I knockdown group (Figures 7a and b). IHC demonstrated reduced ST6Gal-I expression in neoplastic tissue extracted from MHCC97-H/shST6Gal-I mice compared to control animals (Figure 7c). Next, we verified the expression levels of these molecules during DENA-induced liver tumorigenesis by western blotting (Figures 7d and e) and IHC (Figure 7f). Notably, these proteins were significantly increased in the experimental but not in the control groups at 10 and 24 weeks. Therefore, ST6Gal-I might be directly involved in the tumorigenesis and HCC growth via the Wnt pathway.

RETRACTED

## Discussion

Cell surface glycosylation, affecting the interactions between proteins, regulates membrane protein organization.^27^ Abnormal sialylation was found in many cancers, potentially affecting tumor cell differentiation, adhesiveness and invasion.^28^ Here, we examined the expression and localization of ST6Gal-I and sialylation in liver tumor specimens because hepatocytes are known to produce these proteins in large quantities. IHC examination revealed that ST6Gal-I overexpression was higher in HCC tissues of different grades than in to non-tumor liver tissues, and it was secreted into the cytoplasm. Additionally, the IHC results showed that patients with higher ST6Gal-I expression have a lower survival rate. This result is not consistent with that reported by Poon *et al.*,^29^ which may be because their sample size was small, yielding inaccurate results, or because they probably focused on terminal patients, in which ST6Gal-I probably has been already released into the peripheral blood as well as body fluid. Thus, it remains to be explored whether the release of ST6Gal-I from the cytosol into peripheral blood corresponds to increased HCC grade. Experiments such as an enzyme-linked immunosorbent assay are needed to verify our current result, and serum ST6Gal-I levels in patients at different liver cancer stages should be tested. Monitoring of HCC progression using patient blood samples has not yet been achieved.

To explore the role of ST6Gal-I in HCC in detail, we modified its expression in Huh-7 and MHCC97-H cell lines *in vitro*, then aimed to comprehensively elucidate its function during human HCC progression. We found that overexpression of ST6Gal-I enhanced proliferation of HCC cells, increased their migration and invasion *in vitro*, and promoted cell cycle progression, with knockdown of this protein exerting contrary effects. Notably, ST6Gal-I dysregulation is tightly correlated with tumor metastasis. For the *in vivo* xenograft experiment, we employed MHCC97-H cells, which have a higher rate of tumorigenicity than Huh-7 cells, and found that ST6Gal-I knockdown via shRNA reduced tumor volume and growth, confirming the function of ST6Gal-I in promoting neoplasm progression. These findings clearly suggest that ST6Gal-I may positively regulate tumor cell attributes such as proliferation, migration and invasion.

RETRACTED

Hepatocellular carcinogenesis is a complicated process resulting from multiple molecular events leading to the initiation, promotion and progression of tumors.^30, 31^ Zhao *et al.*^32^ reported that sialylation might modulate the invasion and chemosensitivity of HCC, likely through ST6Gal-I or ST8SIA-II regulation of PI3K/Akt signaling. However, to clarify the function of ST6Gal-I in HCC and the associated mechanisms, we examined MAPK, Wnt and PI3K/Akt pathways. ERK signaling plays an important role in the regulation of proliferation, invasiveness and survival in cancers.^33^ However, our results demonstrated that ST6Gal-I upregulation/downregulation did not affect the phosphorylation levels of Erk and JNK. Furthermore, the tumor-cell-surface glycoprotein, EMMPRIN/CD147 (extracellular matrix metalloproteinase inducer) can induce the secretion of matrix metalloproteinases (MMPs) in the tumor–stroma interaction. MMPs are also considered to play major roles in cell processes such as migration, differentiation, angiogenesis and cancer metastasis.^34^ Additionally, the Wnt/β-catenin pathway is also involved in the modulation of tumor angiogenesis and metastasis by affecting the expression of MMP-2 and MMP-9. Our discoveries partly corroborate the supposition that ST6Gal-I can regulate Wnt/β-catenin signaling.

Wnts are N-glycoproteins, and modification of some of them, such as Wnt3a, activates the Wnt/β-catenin canonical pathways.^35, 36^ Binding of the Wnt ligand to the receptor Frizzled-7 promotes the nuclear translocation of cytoplasmic β-catenin, which then associates with TCF/LEF transcription factors, and Frizzled receptors are also N-glycosylated.^37^ These studies indicate that N-glycoproteins play essential roles in Wnt/β-catenin signaling. Our study revealed that ST6Gal-I upregulation led to a significant increase in cytoplasmic β-catenin and release into the nuclear. Furthermore, western blotting demonstrated that related molecules (p-GSK-3β, β-catenin, cyclin D1, c-Myc and MMPs) were significantly decreased in MHCC97-H/shST6Gal-I cells, but increased in Huh-7/ST6Gal-I cells. These findings indicate that ST6Gal-I regulates the Wnt/β-catenin pathway which might be attributed to the modulation of N-glycosylation of Wnt receptors, and Wnt/β-catenin signaling appears to be involved in ST6Gal-I-induced malignant transformation of HCC cells. However, the detailed molecular mechanisms how ST6Gal-I modulates the Wnt signaling pathway are still needed to elucidate in further researches.

RETRACTED

In conclusion, our data implicate that ST6Gal-I overexpression in human HCC is associated with carcinoma progression and poor clinical prognostic. In addition, ST6Gal-I may accelerate HCC development through Wnt/β-catenin signaling. Our findings not only reveals the pathological roles of ST6Gal-I in HCC, but also provide a potential new marker for HCC.

## Materials and methods

### Patients and IHC

ST6Gal-I levels in hepatoma carcinoma and normal hepatic tissues were evaluated by IHC using anti-ST6Gal-I on commercial tissue arrays (Shanghai Zhuo Li Biological Technology, China) as previously described.^38, 39^ After antigen retrieval and blocking, the slides were incubated with a rabbit anti-ST6Gal-I primary antibody (1:100; Abcam, Cambridge, UK) overnight at 4 °C. Negative control slides were processed in the same manner, without addition of the primary antibody. For detection, diaminobenzidine (DAB) (ZSGB-BIO, Beijing, China) and hematoxylin were used. Two certified pathologists blinded to the clinical data independently assessed ST6Gal-I immunostaining, scoring the results depending on the positive-staining percentages and staining intensity, as follows: (0) 0%, no staining (–); (1) 1–29%, weak positive (+); (2) 30–59%, moderate positive (++); and (3) >60%, intense staining (+++). For statistical analysis, cases were categorized as either negative (no and weak staining) or positive (moderate and intense staining). Pearson’s chi-squared test was used to assess the association between ST6Gal-I and HCC, to determine its clinical significance.

### Cell culture

L02 normal liver cells and Huh-7 and MHCC97-H human HCC cells were purchased from the Cell Bank of Chinese Academy of Sciences (Shanghai, China). All cell lines were maintained in Dulbecco’s modified Eagle’s medium supplemented with 10% fetal bovine serum and 1% penicillin/streptomycin under standard culture conditions (37 °C, 5% CO_2_), they were tested regularly for mycoplasma contamination in the laboratory.

### Vector construction and transfection

Huh-7 cells were transfected with the recombinant pcDNA3.1/ST6Gal-I vector or a control vector.^16^ To inhibit ST6Gal-I expression, MHCC97-H cells were transfected with shRNA sequences targeting ST6Gal-I and a negative control vector (shNC) was constructed as described previously.^16, 24^ These cells were transfected with a mixture of plasmids and Lipofectamine 2000 (Invitrogen, Carlsbad, CA, USA) depending on the manufacturer’s instructions. To select stably transfected cells, the culture medium was replaced with complete medium containing 800 mg/ml of G418 (Sigma-Aldrich, Darmstadt, Germany) after 48 h. Modified expression was confirmed by qPCR and western blotting.

RETRACTED

### qPCR

Total RNA was extracted using TRIzol reagent (Life Technologies, Carlsbad, CA, USA) and was employed to synthesize cDNA using a PrimeScript RT Reagent Kit (Takara, Dalian, China) and subsequently mixed with qPCR SuperMix (Takara, Otsu, Japan). Relative changes in gene expression were analyzed using the 2^−ΔΔCT^ method. Sequences of the forward (F) and reverse (R) primers used for qPCR are shown previously.^16^

### Western blot

Proteins were extracted from cells using lysis buffer (Beyotime, Haimen, China) containing protease inhibitors. Protein concentrations in lysates were measured with a BCA kit (Beyotime). Aliquots of protein extracts were subjected to 10–15% SDS–PAGE and then transferred to polyvinylidene fluoride (PVDF) membranes (Pall Corporation, New York, NY, USA), which were blocked for 2 h with 5% skim milk in tris buffered saline, with tween-20 (TBST). The membranes were incubated with primary antibodies of ST6Gal-I (1:600; Abcam, ab77676, Cambridge, MA, USA), PI3K (1:500, Elabscience, ENT3709, Wuhan, China), Akt (1:500, Abcam, ab8805), p-Akt (1:500, Elabscience, ENP0006), GSK-3β (1:500, Affinity Biosciences, AF5016, Cincinnati, HO, USA), phosphorylated Ser9 GSK-3β (1:500, Bioworld, BS4084), β-catenin (1:500, Elabscience, ENT0672), p-β-catenin (1:500, Elabscience, ENP0047), Erk (1:500, Elabscience, EPP12809), p-Erk (1:500, Elabscience, ENP0497), JNK (1:500, Elabscience, EPP14522), p-JNK (1:500, Elabscience, ENP0156), Cyclin D1 (1:500, Affinity Biosciences, DF6386), c-Myc (1:500, Bioworld, BS2462, Louis Park, MN, USA), TCF1 (1:200, Santa Cruz Biotechnology, Inc, Santa Cruz, CA, USA), TCF3 (1:500, Bioworld, BS2466), TCF4 (1:500, Bioworld, P15884), MMP-2 (1:200, Santa Cruz Biotechnology, SC-10736), MMP-7 (1:600, Bioworld, BS1239), MMP-9 (1:200, Santa Cruz Biotechnology, SC-10737), EMMPRIN (1:500, Bioworld) and glyceraldehyde-3-phosphate dehydrogenase (GAPDH) (1:5000; Proteintech, 10494-1-AP, Pearl Street, IL, USA) antibodies. Subsequently, the membranes were incubated with horseradish peroxidase-conjugated secondary antibody (1:10,000; ZSGB-BIO, ZB-2301). Following further washing with TBST, blots were visualized using enhanced chemiluminescence reagents (Advansta, Menlo Park, CA, USA). After exposure, protein band densitometry was conducted with the Image Lab software (Bio-Rad, Hercules, CA, USA).

### Immunofluorescence and confocal microscopy

Cells were plated on slips for 24 h, then these cells were fixed with 4% paraformaldehyde for 30 min, and permeabilized using 0.1% Triton X-100 for 10 min in the dark. They were blocked with 10% bovine serum albumin for 30 min, and incubated overnight with rabbit anti-ST6Gal-I (1:100; Abcam, b77676) and rabbit anti-β-catenin (1:100, Elabscience, ENT0672). A fluorescein-labeled secondary antibody (1:100, Proteintech, SA00006-4) was subsequently incubated with the cells for 1 h at 37 °C. Golgi apparatus were identified using a rabbit anti-GM130 antibody (1:50; BD Biosciences, Franklin Lakes, NJ, USA), and 4,6-diamidino-2-phenylindole was used to stain nuclei for 10 min. Fluorescence was observed using a confocal laser-scanning microscope (BD Biosciences).

RETRACTED

### Soft-agar colony formation assay

0.75% low gelling temperature agarose (Sigma-Aldrich) in complete medium served as the bottom layer, and approximately 4 × 10^4^ Huh-7 or 8 × 10^4^ MHCC97-H cells suspended in 0.36% agarose in the same medium constituted the top layer in 6-cm dishes. After 4 weeks of incubation, the number of colonies with>50 cells in each dish was counted using cellSens software Olympus, Tokyo, Japan).

### Flow cytometry

After washing thrice with phosphate-buffered saline (PBS), cells were collected in a tube, and fixed in 70% cold ethanol overnight. Then, they were blocked with 2% bovine serum albumin and incubated on ice for 30 min with 2 μg/mml fluorescein isothiocyanate (FITCc-onjugated) sambucus nigra agglutinin (SNA). After three washes with PBS, flow cytometry was carried out (FCM, Accuri C6 Cytometer; BD Biosciences, San Jose, CA, USA). The cell cycle distribution of Huh-7/MHCC97-H was analyzed by staining with 50 μg/ml propidium iodide. Finally, 1 × 10^4^ cells from each sample analyzed by FCM.

### Transwell migration and invasion assay

Following the manufacturer’s instructions, serum-free Dulbecco’s modified Eagle’s medium was placed in the upper chambers of a Transwell plate (pore size: 8.0 μm; diameter: 6.5 mm; Corning, NY, USA), and 600 μl complete medium Dulbecco’s modified Eagle’s medium was added to the lower chambers as a chemoattractant. In each well, 8 × 10^4^ Huh-7 or 4 × 10^4^ MHCC97-H cells seeded in the upper chamber and incubated for 32 h. Migrated cells were fixed in 4% paraformaldehyde and stained with 0.1% crystal violet for 30 min, and counted in five non-overlapping fields and photographed. The invasion assay was carried out as above, except that the upper chambers of 24-well Transwell systems were coated with 40 μl Matrigel (diluted 1:8). After 30 min for Matrigel solidification, 1.6 × 10^5^ Huh-7 or 8 × 10^4^ MHCC97-H cells were seeded in each upper chamber and cultured for 48 h.

### Xenograft model

All *in vivo* experiments were approved by and carried out according to the guidelines and regulations of the Dalian Medical University Sciences Center Animal Care and Use Committee. In addition, use of animals in the present study was consistent with Association for Assessment and Accreditation of Laboratory Animal Care International guidelines. Athymic nude mice aged 4–6 weeks were obtained from the Animal Experiment Center of Dalian Medical University, China, for analysis of tumorigenicity. They were randomly divided into three treatment groups, each of which included 10 animals: an MHCC97-H group, a negative control group and an MHCC97-H/shST6Gal-I group. Approximately 2 × 10^7^ cells in 100 μl of PBS were injected subcutaneously into the right dorsal flank of each mouse. Tumor diameters were measured with a vernier caliper every 3 days after 1 week, and tumor volumes being calculated using the following formula: 1/2 (length × width^2^). All mice were killed 30 days later, then tumor weights and volumes were determined. To ascertain the significance of results, the group size was chosen as to ensure that >5 animals remained in each group after 1 month when applying exclusion criteria or if death occurred during the experiment. No statistical method was used to estimate sample size.

RETRACTED

### DENA- and CCl_4_-induced liver tumorigenesis

C57BL/6J mice 6–8 weeks of age weighing 15.8±1.5 g (average±s.d.) were purchased from Dalian Medical University and housed in a temperature-controlled, air-conditioned, specific pathogen-free facility, and received food and water *ad libitum*, taking into consideration the guidelines and regulations of the Dalian Medical University Sciences Center Animal Care and Use Committee. The mice were divided into DENA-treated and control groups, those in the former being injected with 1 mg/kg DENA in sterile 15 ml/kg PBS for 3 weeks, and those in the latter being injected with sterile PBS alone. Then, mice in the DENA group received intraperitone injections of 0.2 ml/kg sterile CCl_4_ diluted in sterile olive oil, twice per week for an additional 21 weeks, while control animals were injected intraperitoneally with PBS. Mice were killed at 0, 2, 4, 8, 9, 10, 16, 18, 20, 22 and 24 weeks after initial treatment to analyze liver neoplasm development. Histopathological examinations to identify liver tumors were performed as described previously.^40^ Allocation of the animals and assessment of the outcome were done without blinding.

### Statistical analysis

Data were analyzed with SPSS 16.0 (SPSS Inc., Chicago, IL, USA), and every experiment was done three times and the results were shown as the mean s.e.±s.d. Student’s *t*-test was used to compare two independent groups of data. Differences were considered significant at *P*-values<0.05.

RETRACTED

## Figures and Tables

**Figure 1:** ST6Gal-I is highly expressed in HCC cells and tumor tissues. (**a**) IHC analysis of ST6Gal-I expression in adjacent noncancerous tissues (ANT) and different grades of HCC tissues (*n*=80). (**b**, **c**) HCC patients with higher expression of ST6Gal-I show worse overall (**b**, **c**) disease-free survival. (**d**, **e**) q-PCR and western blot assays were analyzed for the expression of ST6Gal-I in HCC cell lines and normal human hepatocyte cells. *P<0.05. (**f**) Immunofluorescence data verifying the location of ST6Gal-I in HCC cell lines and normal human hepatocyte cells. Original magnification was × 40.

**Figure 2:** Overexpression of ST6Gal-I contributes to proliferation and metastasis in Huh-7 cells *in vitro*. (**a**, **b**, **d**) Analysis of ST6Gal-I expression in Huh-7 cell transfected with pcDNA3.1/ST6Gal-I by qPCR (**a**), western blotting (**b**) and immunofluorescence (**d**). (**c**, **e**) α2, 6-linked sialic acid expression levels determined by lectin blotting and flow cytometry. (**f**) ST6Gal-I overexpression enhances the viability of Huh-7 cells as indicated by CCK-8 assay. (**g**) Colony formation assay was used to evaluate the proliferation of Huh-7 cells after stimulating the expression of ST6Gal-I. (**h**) Cell cycle distribution analysis by FACS showed that the rate of S phase was higher in Huh-7/ST6Gal-I cells than in the control group. (**i**) Migration behaviors of Huh-7 cells with upregulated ST6Gal-I expression explored by a wound-healing assay. (**j**, **k**) Transwell assays showed that overexpression of ST6Gal-I increases the invasion and migration rates of Huh-7 cells. All quantitative data are shown as the mean±s.d. of three independent experiments. *P<0.05.

**Figure 3:** Depletion of ST6Gal-I in MHCC97-H cell line inhibits cell growth and metastasis *in vitro*. (**a**, **b**, **d**) Analysis of ST6Gal-I expression in MHCC97-H cells transfected with shST6Gal-I by qPCR (**a**), western blotting (**b**) and immunofluorescence (**d**), original magnification was × 40. (**c**, **e**) Knockdown of the expression of ST6Gal-I could affect α2, 6-linked sialic acid expression levels as determined by lectin blotting and flow cytometry assay. (**f**) Cell Counting Kit (CCK-8) assays showed that knockdown of ST6Gal-I expression leads to inhibition of cell proliferation. (**g**) Colony formation numbers was lower in ST6Gal-I-low expression cells (MHCC97-H/shST6Gal-I group) than in controls. (**h**) Flow cytometry assay showed that ST6Gal-I depletion leads to G1 arrest. (**i**) Cell migration ability as analyzed by wound healing assay in MHCC97-H cells following ST6Gal-I silencing at different time points. (**j**, **k**) Transwell assays were used to analyze the invasion and migration abilities of MHCC97-H transfected with shST6Gal-I. *P<0.05.

RETRACTED

**Figure 4:** ST6Gal-I promotes liver tumorigenicity in mice. (**a**, **b**) Morphological images of tumors formed after 30 days; representative results are shown. (**c**, **d**) Average tumor weights and sizes were measured in different groups. *P<0.05. (**e**, **f**) Differential expression of ST6Gal-I in the experimental group, negative control group and matched group as examined by IHC and western blot analysis. *P<0.05. (**g**, **h**) IHC and western blot analysis showed that ST6Gal-I expression significantly increases during different periods of DENA-induced liver tumorigenesis.

**Figure 5:** Upregulation of ST6Gal-I activates PI3K/Akt, and Wnt/β-catenin signaling pathways in Huh-7 cells. (**a**, **c**, **e**) Main protein components of the PI3K/Akt/MAPK/β-catenin signaling pathway in Huh-7 cells were measured using western blotting. (**b**, **d**, **f**) Relative protein intensities were determined with the Image Lab software (Bio-Rad). *P<0.05. (**g**) Immunofluorescence imaging analysis was used to monitor β-catenin release from the cytosol into the nuclear space upon overexpression of ST6Gal-I; representative figures are shown. The error bars represent the s.d. of the mean values obtained from triplicate experiments. *P<0.05.

**Figure 6:** Knockdown of ST6Gal-I inhibits PI3K/Akt, and Wnt/β-catenin signaling pathways in MHCC97-H cells. (**a**, **c**, **e**) Main protein components of the PI3K/Akt/MAPK/β-catenin signaling pathway in MHCC97-H cells were measured using western blotting. (**b**, **d**, **f**) Relative protein intensities were determined using Image Lab software. Error bars represent s.d. *P<0.05. (**g**) Subcellular localization of β-catenin in MHCC97-H cells treated with shST6Gal-I plasmids, examined by confocal microscopy. Cells with typical morphology are presented.

**Figure 7:** Altered expression of ST6Gal-I affects liver tumorigenesis via the Wnt/β-catenin signaling pathway in mice. (**a**, **c**) Western blotting and IHC were used to detect the expression levels of GSK-3β, p-GSK-3β, β-catenin, p-β-catenin, Cyclin D1 and c-Myc proteins in tumor tissues. (**d**, **f**) Western blotting and IHC analyses revealed differential expression of these proteins in liver tumorigenesis. (**b**, **e**) Relative protein intensities as determined by Image Lab. *P<0.05.

**Table 1:** Distribution of characteristics of patients with HCC by ST6Gal-I expression

*Patient characteristics*	*ST6Gal-I expression*		*Total*	P *Value*
	*Low*	*High*		
Age, years				0.133
>50	11	27	38	
⩾50	19	23	42	
Sex				**0.023**
Male	21	45	66	
Female	9	5	14	
Number of lesions				**0.014**
Unifocal	18	16	34	
Multifocal	12	34	46	
Serum AFP (mg/l)				0.635
>20	8	11	19	
⩾20	22	39	61	
Extent of invasion				0.515
T1–T2	13	18	31	
T3–T4	17	32	49	
Pathologic grade				**0.021**
I–II	14	11	25	
III–IV	16	39	55	
Lymph node metastases				0.905
Negative	28	47	75	
Positive	2	3	5	

Abbreviations: AFP, alpha fetoprotein; HCC, hepatocellular carcinoma. *P*<0.05 was statistically significant.
